# The Integrated Sustainable Development Mechanism of Sports Industry Based on Recombination Fusion Mode

This article has been retracted.

**DOI:** 10.1155/2022/6906467

**Published:** 2022-06-28

**Authors:** Bo Zhao, Jianmin Chen, Tao Song

**Affiliations:** ^1^Institute of Physical Education, Sichuan University of Science & Engineering, Zigong 643000, Sichuan, China; ^2^Wenzhou Polytechnic, Wenzhou 325035, Zhejiang, China

## Abstract

Regular competitions on a bigger size and level are referred to as sports events. The World Cup, the Olympics, Formula, the NBA, and many intercontinental sports events and World Championships of various individual sporting organizations, among others, are among the world's largest and most significant sporting events. In China, there are also specific live sporting event websites that broadcast weekly sporting events. The purpose of this paper is to study the integrated development mechanism for the sustainable development of natural ecotourism and sports events. For this reason, this paper proposes research and analysis on its industrial integration method and industrial integration path, and it has an in-depth understanding of the sustainable development model. At the same time, relevant experiments are designed in the experimental part to explore the impact of sports events and natural ecotourism in the development process. The experimental results of this paper show that after the improvement, the attractiveness of tourists has increased by 47.48%, which has effectively promoted the development of the related tourism industry.

## 1. Introduction

In essence, leisure sports use people's leisure time in the form of sports activities, so that people can achieve the purpose of leisure. After entering the 21^st^ century, people pay more attention to the body. The demand for leisure is more intense, and the development prospect of leisure sports is bright. If one looks at leisure sports as an industry, there are many paths for its development, however, it has a particularly close relationship with the tourism industry, and it is more suitable for the integrated development of these industries.

In recent years, China's leisure sports industry and tourism industry have achieved rapid development and have a preliminary foundation for the development of industrial integration. Through relevant research, it can play a reference value for the local government's sports tourism development work. This topic will theoretically discuss the relationship between “sports events” and “tourism,” which can enrich the theoretical basis of this field to a certain extent.

The innovation of this paper is to focus on the industrial integration of natural ecotourism and sports events, supplemented by the sustainable development of ecotourism to explore the relevant factors in the process of industrial integration, and to study and improve its future development mechanism, so that the improved industrial integration development mechanism can be more attractive.

## 2. Related Work

With the continuous improvement of people's living standards, the way people travel abroad is becoming more diverse, and the sustainable development of natural ecotourism and the industrial integration of sports events have also attracted more people's attention. Zhang et al. suggested that ecotourism and off-road recreational activities may pose a threat to wildlife inhabiting protected areas. They investigated the flight response patterns of blue sheep living in the Helan Mountains National Nature Reserve in Ningxia, China. It was found that the flight start distance and final flight distance varied within the protected area and were a function of the tourism level of each key area [1]. Baum et al. argues that an important challenge in analyzing cultural services is understanding the geography of service delivery in relation to human and ecosystem elements. He used access rates and context, content, connectivity, and location measurements of 64 private land reserves to better understand the impact of geography on the delivery of cultural services [2]. Dhami et al. emphasized the importance of sensitivity analysis of standard weights when mapping NBT regions in West Virginia. As an extension of the study by Dhami, Deng, Burns, and Pierskalla, they examined and mapped the NBT region of West Virginia by incorporating tourists' perceptions as standard weights into a spatial suitability model [3]. Xu et al. used a choice experiment to explore the trade-offs between ecological protection and leisure services for tourists in Zhalong National Nature Reserve in Northeast China and added socioeconomic and attitude factor analysis to reveal the heterogeneity of preferences. The results show that biodiversity is the most valuable attribute, and increasing biodiversity or/and environmental education facilities is a valuable scenario for wetland development [4]. Ibarra-Michel et al.'s research aims to describe participatory processes and community management and benefits from ecotourism based on the literature reviewed. In this regard, sanctuary defines a case study using a qualitative approach. Semistructured interviews were used to discover community members' perceptions of management participation and the benefits of ecotourism [5]. Shi et al. argues that although new models are needed to address the challenges of managing contemporary protected area systems, large-scale park visitor symbiosis remains an aspiration. However, a survey of 1,050 tourists in northeast China's Hongtan National Scenic Corridor shows potential. According to the claim to adhere to basic ecotourism, 36.0% of the people meet the qualifications of “passionate ecotourists” and “ecotourists” [6]. Using a community capital framework with a systems thinking perspective, Stone and Nyaupane explore how the development of ecotourism affects changes in community needs and, in turn, the functioning of protected areas. The Chobe Enclave Conservation Trust, located near Chobe National Park in Botswana, provided the background for the study, using data collected through semistructured interviews and secondary sources [7]. Bae believes that the concept of cultural services as one of ecosystem service functions, because of the relationship between ecotourism and cultural services, i.e., emphasizing the material and spiritual benefits that human beings obtain from nature, is attracting more people's attention. In addition, from the perspective of cultural services, the quality of human life can be improved through ecotourism. Hence, various basic research data with ecotourism as an indicator of cultural services is needed [8]. The mentioned documents describe the sustainable development of related natural ecotourism in great detail. For the relevant ecological protection issues, there is a more detailed study, however, there is no content that combines sports events and natural ecotourism, and the relevant research depth is not enough.

## 3. Industrial Convergence Approach

### 3.1. Integration of Natural Ecotourism and Sports Industry

#### 3.1.1. The Path of Industrial Integration and Development

The word “path” comes from the concept of geography, and now, it mostly refers to the path from the starting point to the end point. Starting from the origin of the word “path,” this paper redefines the path of the integration of natural ecotourism and sports industry (the ways and means to realize the integrated development of natural ecotourism and sports industry). The integration of tourism and sports industry, as a multilevel and multicontent integration process, not only has a general integration path but also has its own characteristics [9].

#### 3.1.2. Penetration of Sports Industry into Tourism Industry

The form in which the sports industry penetrates into the tourism industry is mainly the packaging and marketing of three sports industry resources, such as competition performances, leisure sports, and sports training bases, to be transformed into tourism products [10]. The fusion mode for penetration is shown in Figure 1.

With the continuous improvement of the economic level, people's living conditions are increasingly abundant, and more people are beginning to pursue a high-quality life. This demand of people has brought a huge market space for leisure fitness tourism [11]. The main items of leisure fitness include rock climbing, bungee jumping, skiing, swimming, and so on. It can broaden the horizons, broaden the breadth of tourism activities, and increase the tourism attraction of each representative city with the help of rich regional resources in the planning and development of leisure and fitness projects.

#### 3.1.3. Industrial Integration of Natural Ecotourism and Sports Events

Industrial integration is a process in which the industrial outlines of several industries are clearly defined, gradually become unclear, and finally disappear. Before the integration of tourism industry and sports industry, they provide products for industries within the border through self-sufficiency. With the continuous innovation of various industries, new products are born because of the integration of the two industries spanning, and consumer demand increases [12]. Since this moment, the outline of the industry has become no longer clear. With the continuous improvement of integrated products, new industrial forms have finally become dominant, new industries have been generated, and industrial integration has been realized. The realization process of industrial integration is shown in Figure 2.

The natural ecotourism industry and the sports industry are developing rapidly, and the integrated development of industries has become an inevitable trend in the economic development of this model. The integrated development of the two industries can realize the diversification of tourism products and promote the industrialization of the sports industry with the help of the tourism platform. A variety of factors promote the integration of industries, and the reasons for the integration of natural ecotourism and sports industry mainly include the subsequent three aspects [13, 14].

*(1) Advancedization of Consumer Demand*. The input of sports resources can enrich the products and forms of tourism, thus forming characteristic sports tourism activities. At the same time, because of its unique function (leisure and entertainment, physical fitness, and enriching life content), sports activities enable people to not only enjoy the beautiful scenery but also participate in various activities (physical exercise, sports events, sports adventure, and sports cultural exchange) to achieve the purpose of pleasing body and mind.

*(2) Changes in Market Supply*. With the continuous improvement of residents' living standards, people begin to pursue higher-level and richer tourism products and sports products more urgently, requiring changes in the supply content of enterprises.

*(3) Continuous Innovation of High Technology*. Technological innovation has brought support for the integration and upgrading of tourism and sports industry in Hebei Province, and it is the medium and link of the integration of tourism and sports industry. The great development of information technology shortens the distance between tourists and the destination, enhances the ability of information communication, and strengthens the market connection, which makes tourism activities more convenient. At the same time, the development of technology also reduces the cost of products and makes products more accessible.

*(4) The Penetration of Tourism Industry into Sports Industry*. The way the tourism industry penetrates into the sports industry is mainly to actively integrate sports elements in multiple links of tourism products (design, production, sales, and service links). The abundance of tourism resources, diverse forms, and beautiful natural scenery determine the content, form, and scale of sports activities and also provide excellent venues and resources for sports activities [15, 16].

Compared with the state in the permeable fusion model, the reorganization and fusion model realizes the innovation of the industrial form, and new forms of business appear. This phenomenon generally occurs in different industries in the same industry or in closely related industries. New products or services are produced in the process of integration. In the process of the re-integration of tourism and sports industries, platforms are built by means of exhibitions, festivals, industrial gathering parks, characteristic projects, and other factors, thus forming four new tourism formats. As shown in Figure 3, the development of these four formats is not the same.

*(5) Extended Industrial Integration*. In the integration mode of natural ecotourism and sports industry integration, the extension-type industrial integration is different from the penetration-type and reorganization-type integration, and it requires more preconditions to be completed. First of all, the tourism and sports industries are required to have a functional complementary relationship, which is mainly reflected in economic activities, and they also need to have the ability to extend the role of economic activities. The industrial chain of the industry itself will have a certain degree of extension, and the realization of integration will take place in this part. In this part of the extension, the boundary will gradually weaken, and a new fusion industry will be generated through the form of intersection. Through this function, the original functions are expanded and new added value is generated, thereby obtaining new and stronger core competitiveness [17]. At the same time, the direction of the extended integration of natural ecotourism and the sports industry is also different from the two-way penetration of the permeable type, which is a single extension of the sports industry to the tourism industry. The attributes of the sports industry determine that it has a strong ability to extend and can be extended to related industries, as shown in Figure 4 by extending to other industries.

The extension and integration of the tourism and sports industries is the result of the mutual development and mutual promotion of the two industries, which promotes the development of new formats. From the perspective of the development status of the sports industry, the five industry formats formed by the extension of the core sports industry, whether it is the development of sports culture and creative industry, sports-themed bar and catering industry, outdoor sports equipment manufacturing, sports betting industry, and the development of characteristic sports tourism industry R&D centers, belong to the blank or budding stage, and tourism products combined with tourism elements are even more difficult.

“Creativity” and “Science and Technology,” as weak links in industrial development, seriously restrict the integrated development of tourism and sports industry. Proceeding from the actual situation, it is difficult to realize the extension-type integration mode, and the conditions for the integration of various extension industries are not satisfied and immature. Identifying the industry chain with the sports industry, integrate the extension of the sports industry chain with the tourism industry, and integrate in an appropriate way to accurately grasp the method and entry point [18].

### 3.2. The Benefit Distribution Mechanism of the Coupling System between the Sports Industry and the Tourism Industry

When the sports industry and the tourism industry build a coupled system, the coupled system will encounter a problem, i.e., how to distribute the benefits, and the distribution of benefits affects the development of the coupled system of the tourism industry and the sports industry [19]. To realize the sustainable development of the coupled system, a fair and scientific benefit distribution mechanism must be established to provide a guarantee for the development of the coupled system. This section establishes a game model for the benefit distribution of the coupled system and analyzes the problems in the benefit distribution of the tourism and sports industries after they are coupled [20].

When distributing the coupling benefits of the tourism industry and the sports industry, the organization that manages the tourism industry is *A*_2_, and the organization that manages the sports industry is *A*_1_. The sports industry department and the tourism industry management agency manage the coupling system according to the industry under their jurisdiction [21]. *e*_1_ is the contribution made by the organization managing the sports industry to the coupling system, and *e*_2_ is the contribution made by the organization managing the tourism industry to the coupling system. At this time, the output is expressed by the following formula:

(1) $$\begin{array}{c} Y=f\left(e_{1},e_{2}\right)+\xi . \end{array}$$

In the coupled system, both the agencies that manage the tourism industry and the agencies that manage the sports industry have made certain contributions, which shows that *e*_1_ and *e*_2_ have a complementary relationship. Hence, the increasing concave function of the contributions made by the two governing bodies is the system output.

In the sports and tourism industry coupling system, the sports industry competent department and the tourism industry management agency distribute the output of the coupling system. To make the calculation more concise, *a*_1_ is used to represent the contribution coefficient of the organization that manages the sports industry, and *a*_2_ is used to represent the contribution coefficient of the organization that manages the tourism industry. The random variable is represented by *ξ*. At this time, the output function can be expressed as follows:

(2) $$\begin{array}{c} Y=\left(a_{1}e_{1}+a_{2}e_{2}\right)+\xi . \end{array}$$

Among them, *ξ* is a random variable, obeying *N*(0,2).

The effort cost of *A*_1_ and *A*_2_ can be equivalent to the monetary cost. Then, the effort cost of the two competent departments in the coupled system of sports industry and tourism industry is as follows:

(3) $$\begin{array}{c} C_{i}\left(e_{i}\right)=C_{i}+\frac{1}{2}\gamma_{i}e_{i}^{2}. \end{array}$$

In the coupling system of sports industry and tourism industry, the distribution of interests between the competent departments of sports industry and tourism industry is the output sharing mode. In the coupled system, the institutions that manage various industries obtain their own benefits according to the relevant proportions. They share the benefits together, and at the same time, they also bear certain risks.

#### 3.2.1. Construction of the Model

According to the assumptions, the actual income of the sports and tourism industry coupling system, the actual income of the sports industry competent department *A*_1_, and the actual income of the tourism industry competent department *A*_2_ can be calculated as follows:

(4) $$\begin{array}{c} \pi =Y-C_{1}\left(e_{1}\right)-C_{2}\left(e_{2}\right),\\ \pi_{A_{1}}=sY-C_{1}\left(e_{1}\right),\\ \pi_{A_{2}}=\left(1-S\right)Y-C_{2}\left(e_{2}\right). \end{array}$$

Considering the risks in the coupling system of the sports industry and the tourism industry, the deterministic equivalent income of the entire coupling system can be obtained as follows:

(5) $$\begin{array}{c} E\pi -C_{A_{1}}-C_{A_{2}}=Y-\left[C_{A_{1}}+C_{1}\left(e_{1}\right)\right]-\left[C_{A_{2}}+C_{2}\left(e_{2}\right)\right], \end{array}$$

(6) $$\begin{array}{c} E\pi_{A_{1}}-C_{A_{1}}=sY-\left[C_{A_{1}}^{2}+C_{1}\left(e_{1}\right)\right], \end{array}$$

(7) $$\begin{array}{c} E\pi_{A_{2}}-C_{A_{2}}=\left(1-S\right)Y-\left[C_{A_{2}}+C_{2}\left(e_{2}\right)\right]. \end{array}$$

According to the formula, the members of the coupling system established by the tourism industry and the sports industry formulate cooperation strategies according to the goal of maximizing interests. The optimal effort level of sports industry authorities and tourism industry authorities in a coupled system under Pareto equilibrium is as follows:

(8) $$\begin{array}{c} \frac{\partial \left(E\pi -C_{A_{1}}-C_{A_{2}}\right)}{\partial e_{1}}=a_{1}-\gamma_{1}e_{1}=0,\\ \frac{\partial \left(E\pi -C_{A_{1}}-C_{A_{2}}\right)}{\partial e_{1}}=a_{1}-\gamma_{2}e_{2}=0. \end{array}$$

The maximum level of effort for agencies managing the tourism industry and managing the sports industry is as follows:

(9) $$\begin{array}{c} e_{1}^{0}=\frac{a_{1}}{\gamma_{1}},\\ e_{1}^{0}=\frac{a_{2}}{\gamma_{2}}. \end{array}$$

**Conclusion 1 .**

In the coupling system of sports industry and tourism industry, there is a positive correlation between the efforts and contribution coefficients of the organizations that manage the tourism industry and the organizations that manage the sports industry to maximize the benefits, and the coefficients of their own variable costs are negatively correlated.

In the coupling system of the sports industry and tourism industry, the agencies that manage the tourism industry and the agencies that manage the sports industry have formulated a noncooperative strategy to maximize profits. Under Nash equilibrium conditions, the optimal effort level of the agencies that manage the tourism industry and the agencies that manage the sports industry is as follows:

(10) $$\begin{array}{c} \frac{\partial \left(E\pi -C_{A_{1}}\right)}{\partial e_{1}}=sa_{1}-\gamma_{1}e_{1}=0,\\ \frac{\partial \left(E\pi -C_{A_{1}}\right)}{\partial e_{2}}=\left(1-s\right)a_{2}-\gamma_{2}e_{2}=0. \end{array}$$

According to the formula, it can be understood that the maximum level of effort made by the institutions that manage the tourism industry and the management of the sports industry is as follows:

(11) $$\begin{array}{c} e_{1}^{*}=\frac{sa_{1}}{\gamma_{1}}, \end{array}$$

(12) $$\begin{array}{c} e_{1}^{*}=\frac{\left(1-s\right)a_{2}}{\gamma_{2}}, \end{array}$$

(13) $$\begin{array}{c} \frac{e_{1}^{*}}{e_{2}^{*}}=\frac{s}{1-s}\cdot \frac{a_{1}}{a_{2}}\cdot \frac{\gamma_{2}}{\gamma_{1}}. \end{array}$$

**Conclusion 2 .**

In the coupling system of sports industry and tourism industry, there is a positive correlation between the level of effort made by the competent departments of the sports industry and the competent departments of the tourism industry when they pursue their own maximum interests and the benefit distribution coefficient. The relationship with the contribution coefficient is a positive correlation, and the relationship with the variable cost coefficient is a negative correlation, which is consistent with reality. Hence, the aforementioned assumptions are consistent with reality.

According to formulae (11) and (12), we obtain the following:

(14) $$\begin{array}{c} \frac{\partial e_{1}^{*}}{\partial s}=\frac{a_{1}}{\gamma_{1}},\\ \frac{\partial e_{2}^{*}}{\partial s}=\frac{a_{2}}{\gamma_{2}}. \end{array}$$

It can be obtained from formula (5) as follows:

(15) $$\begin{array}{c} \frac{\partial \left(E\pi -C_{A_{1}}-C_{A_{2}}\right)}{\partial e_{1}}=a_{1}-\gamma_{1}e_{1}=0,\\ \frac{\partial \left(E\pi -C_{A_{1}}-C_{A_{2}}\right)}{\partial e_{2}}=a_{2}-\gamma_{2}e_{2}=0. \end{array}$$

**Conclusion 3 .**

There is a positive correlation between the distribution coefficients and contribution coefficients of various subjects in the coupling system of the sports industry and tourism industry. When the contribution coefficient becomes larger, the distribution coefficient will also increase. The relationship between the distribution coefficient and the variable cost coefficient is a negative correlation. When the variable cost coefficient expands, the distribution coefficient will become smaller. It can be seen that as far as various subjects in the coupled system are concerned, if they play a more important role, their contribution coefficient is larger, or when the variable cost coefficient is small, they have an advantage in distributing benefits, and their coefficient of sharing benefits is also large [22].

General researchers believe that the benefit distribution mechanism must make the risks shared by the subjects in the coupled system proportional to the benefits obtained, which enables each subject in the system to work actively and reflects the principles between systems (i.e., sharing the benefits together, taking the risks together, and sharing the investment together) [23]. However, in the coupled system, the agencies that manage the tourism industry and the sports industry are in a competitive and cooperative relationship with each other, and there are quasi-excess returns in the coupled system. Hence, in this system, whichever management agency can take advantage of, it should pay attention to the temptation of default by the more disadvantaged authorities, otherwise, members of the coupled system may implement opportunistic behavior. To eliminate breaches, punishment or incentives are usually used. However, the coupled system is a loose organization. In addition to establishing a formal organizational mechanism, some informal organizational mechanisms should also be used to provide guarantees for the operation of the coupled system.

### 3.3. Sustainable Development of Ecotourism

According to the meaning of sustainable development, the sustainable development of ecotourism can be generally understood as meeting the needs of contemporary tourists and destination residents while maintaining and enhancing future development opportunities through the sustainable management of existing tourism resources, ensuring stable operations in many aspects (cultural integrity, basic ecological processes, biodiversity, and life support systems) to maximize the economic, social benefits, and aesthetic needs of eco-tourism. Specifically, the sustainable development of ecotourism mainly includes the following meanings and requirements:

#### 3.3.1. The Sustainable Development of Ecotourism Is First Manifested in the Maintenance of the Sustainable Development of Natural Ecosystems

The object of ecotourism is mainly a relatively complete natural ecosystem. Therefore, the sustainable development of natural ecosystems will inevitably become the main content of the sustainable development of ecotourism. A good and rich natural ecological environment is the destination of ecotourism. Natural ecosystems do not tolerate any depleting consumption. Therefore, whether it is business developers, management decision makers, or tourists, they have an inescapable responsibility for protecting the natural ecological environment. It is necessary to understand and protect nature in the practice of ecotourism. This kind of ecological protection includes not only the normal development of natural ecosystems and the maintenance of cyclic stability but also the maintenance of the harmonious coexistence between human and nature, i.e., respect for the local culture. This responsibility for respecting and protecting the tourist objects is an important connotation of the sustainable development of ecotourism.

#### 3.3.2. The Sustainable Development of Ecotourism Includes the Purpose of Promoting Tourism Areas and Sustainable Development

Promoting the sustainable economic and social development of ecotourism is an important purpose of ecotourism, which is embodied in two levels: the individual level of the residents of the tourism destination and the overall level of the tourism destination's society, economy, and culture. Residents of tourist destinations are an important part of tourism society and culture, and they have the right to maintain their own sound development. Therefore, the development of ecotourism must involve the direct participation of local residents in management services. From the perspective of environmental impact, the maintenance and impact of local residents on the natural environment is more direct than that of tourists. In a word, the development of ecotourism makes it possible for local residents to protect resources scientifically, economically, and technically. From an economic point of view, such participation enables them to obtain rich economic returns and effectively promote the economic development of tourist destinations. From the perspective of social development, the development of tourism in the local area has broadened their horizons, improved their quality, and integrated into modern civilization more quickly.

#### 3.3.3. Framework Analysis of Sustainable Development of Ecotourism

The sustainable development system of ecotourism is the intersection of economic system, ecological system, and social system, and it involves various fields of ecological economy, ecological society, and social economy. Therefore, the sustainable development goals to be achieved by ecotourism should be achieved simultaneously with the three-dimensional goals of economy, society, and ecological environment. Its implementation mode is shown in Figure 5.

Starting from the figure, the sustainable development goals of ecotourism are divided into components, namely the main body of ecotourism—ecotourists, objects—ecotourism resources, media—ecotourism enterprises, and carriers—ecotourism environment. From this, the thinking target mode of ecotourism is constructed, as shown in Figure 6.

## 4. Experiment on the Interactive Development of Sports Events and Urban Tourism

Existing studies have pointed out that the interactive development of large-scale sports events and urban tourism at the demand level are conducive to meeting the publicity needs of large-scale sports events and can promote the development of urban tourism. Obviously, tourism companies have a large number of regular urban tourism customers. They can expand the popularity and attractiveness of events by promoting their event tourism products, and through the reception and service guarantee provided by tourism-related enterprises, to a certain extent, it can enhance tourists' trust in sports event tourism and enhance the tourism appeal of sports events.

To this end, on the basis of analyzing the literature data, this paper also conducts a questionnaire survey of experts on this issue. The statistics are shown in Table 1:

As can be seen from the table, the vast majority of the interviewees believe that holding sports events has an impact on the development of urban tourism, and only 25% of the interviewees believe that sports events do not necessarily have an impact on urban tourism. This statistical result is basically consistent with the results obtained by a large number of literature studies, and most scholars and experts agree that sports events have a certain impact on urban tourism. This survey result not only proves the feasibility of the remaining questions of this questionnaire but also is the premise guarantee for the follow-up research of this paper to continue. At the same time, this paper investigates and studies the impact of large-scale sports events on urban tourism. The survey results are shown in Table 2.

As shown in the table, 41.7% of the respondents believe that sports events have a very important and relatively important impact on urban tourism, only 8.3% of the respondents believe that sports events have only a generally important impact on urban tourism, and only one interviewee believes that sports events have a less important impact on urban tourism. It can be seen from the table that the vast majority of respondents believe that sports events have a certain degree of influence on urban tourism, accounting for 90% of all respondents. To sum up, the influence of holding large-scale sports events on urban tourism is basically recognized, and its influence is relatively significant.

As known, the impact of holding large-scale sports events on urban tourism is often multidimensional, and its positive impact will also be reflected in many aspects. In the previous literature analysis, this research classified and compared one by one and finally divided the main impact of large-scale sports events on urban tourism into five categories. This paper conducts a questionnaire survey on the impact of these five aspects. The first is the impact on the tourism economic index, which mainly includes the impact on the number of tourists, tourism revenue, and tourism foreign exchange. The second is the impact on tourism hardware facilities, such as the hardware facilities of hotels, restaurants, and other supporting enterprises. The third is the impact on the soft power of the tourism industry, mainly including the level of tourism reception services. The fourth is the structural impact on tourism, such as the impact on the structure of tourist sources, the structure of tourism off-peak seasons, and so on. The fifth is the impact on urban tourism and cultural exchanges, and the survey results are shown in Table 3.

To verify the impact of sports events on the urban tourism economy, this study investigates this issue. The survey results are shown in Table 4.

Scholars are still divided on the impact of major sporting events on the number of tourists in host cities, the view that it can increase the number of tourists, and the view that it will reduce the number of tourists. While these views coexist, most studies support that large-scale sporting events can increase the number of tourists to the event host city to a certain extent. Therefore, this study investigates this issue. The survey results are shown in Table 5.

The results of this survey show that most of the respondents believe that it is necessary to evaluate the impact of large-scale sports events on the number of tourists. It should be analyzed according to the specific event and the impact of different levels, and the scales of events on the number of tourists is not the same.

## 5. The Integration of Ecotourism and Sports Events Industry

### 5.1. ARMA Forecast and Analysis of Sustainable Development of Tourism Industry

Sustainable development is a dynamic process. It is necessary to study not only the past and current development stage of the region but also the sustainable development trend of tourism in the future. To scientifically display the laws and trends of sustainable tourism development, providing a quantitative basis for the formulation of regional tourism development plans and policies, it is of great significance to the sustainable development of regional tourism. Therefore, this paper uses the ARMA forecast model to analyze the sustainable development trend of tourism in city A from 2006 to 2015 to predict the sustainable development trend of tourism in the future to 2025 under the current scenario conditions.

Firstly, the tourism income of city A from 2006 to 2015 is set as a continuous time series, and the ADF unit root test is carried out to test the stationarity of the series using Eviews9.0 software. The autocorrelation and partial correlation analysis are carried out. Five models of ARMA (1, 0), ARMA (2, 0), ARMA (1, 1), ARMA (1, 2), and ARMA (1, 3) were established and using the residual sequence and AIC of the regression results, SC and R2 are tested. It is concluded that ARMA (2, 0) is the optimal model, which can be used for predictive analysis. The result is shown in Figure 7.

As can be seen from the figure, the predicted value is a gradually rising smooth curve, which is roughly the same as the actual value and has a high degree of fit. In the next 10 years, the overall tourism revenue of city A will continue to rise, reaching the peak in the forecast period in 2022. After 2020, the upward trend of tourism revenue will slow down or even decline.

### 5.2. Prediction and Analysis of Tourism Environment Load Rate ARMA

Firstly, set the 2006–2015 tourism environmental load rate as 0.50, 0.51, 0.51, 0.52, 0.57, 0.59, 0.52, 0.49, 0.61, 0.97, 0.49 as a continuous time series. Use Eviews9.0 software to conduct ADF unit root test for sequence stationarity, and conduct autocorrelation and partial correlation analysis. Three models of ARMA (1, 0), ARMA (1, 0), and ARMA (1, 1) were established, and the serial correlation of the residuals of the regression results, AIC, SC, and adjusted R2 were tested. It is concluded that ARMA (1, 1) is the optimal model, which can be used for predictive analysis. Its prediction model is shown in Figure 8.

It can be seen that the predicted value is a gradually rising smooth curve, which is roughly the same as the actual value, and the fitting degree is good. From 2006 to 2010, city A consumed a large number of nonrenewable resources, produced waste pollution, and seriously affected the regional ecological environment. The environmental load rate of the year dropped significantly compared with the previous year, which was lower than the forecast value for the same period. After 2010, city A has increased its efforts to develop and rectify tourism and paid attention to the protection of the ecological environment in the study area. Therefore, the ARMA model prediction of environmental load rate is feasible. In the next 10 years, the overall load rate of tourism environment in city A will continue to rise. In 2020–2023, the growth rate of the predicted value will reach the highest in the forecast period, and after 2020, the upward trend of the tourism environmental load rate will slow down.

### 5.3. Prediction and Analysis of Tourism Emergy Exchange Rate ARMA

Firstly, set the tourism revenue of city A from 2006 to 2015 as 1.26, 1.27, 1.38, 0.47, 0.81, 1.65, 1.94, 2.49, 2.84, 3.13, 3.81 as a continuous time series. Use Eviews9.0 software to conduct ADF unit root test for sequence stationarity, and conduct autocorrelation and partial correlation analysis. Establish the five models of ARMA (1, 0), ARMA (1, 0), ARMA (1, 1), ARMA (1, 2), and ARMA (2, 1), and test the residual series correlation of the regression results, AIC, SC, and adjusted R2. It is concluded that ARMA (1, 1) is the optimal model that can be used for predictive analysis. Its prediction model is shown in Figure 9.

The predicted value is a gradually rising smooth curve, which is roughly the same as the predicted trend of the actual value, and it has a high degree of fit. In 2008, because of the global economic crisis, the Wenchuan earthquake and the “3.14” event in Tibet, the tourist destination market was affected, the number of tourists decreased sharply, the decrease of tourism input was greater than that of tourism output, and the exchange rate of tourism energy in the current year decreased significantly compared with the previous year, which was lower than the forecast value for the same period. In the next 10 years, the exchange rate of tourism energy in city A will continue to fluctuate and rise as a whole, indicating that the tourism industry is developing well with the support of new technology and has a higher input-output efficiency.

### 5.4. Development before and after the Integration of Natural Ecotourism and Sports Events Industry

To make a comparative analysis of the situation before and after the integration of natural ecotourism and sports events industry proposed in this paper and how to get a general grasp of the specific effect, this paper conducts a simulation experiment on it by conducting experiments on 5 places with roughly the same traffic flow and traffic volume by conducting a statistic on the number of people who experience it to reflect this specific effect. The statistics are shown in Figure 10.

Through the development of the industry before and after the integration in the figure, the attractiveness to tourists before the integration is 31%, 39%, 34%, 26.3%, and 25.2%, respectively. In contrast, after industrial integration, the attraction to tourists is 76%, 83%, 77%, 75.7%, and 81.2%. It can be seen that the improvement is still more obvious.

Based on the analysis, it can be seen that after the industrial integration of natural ecotourism and sports events, the attraction to tourists has increased by 47.48%, and its sustainable development trend has also been significantly improved, which can better promote the tourism industry.

## 6. Conclusions

This article mainly studies the sustainable development of natural ecotourism and the industrial integration of sports events. First of all, the article researches and analyzes the industrial integration of natural ecotourism and sports events, understands the integration situation, and then makes a detailed understanding of the benefit distribution mechanism of the coupling system in the process of industrial integration. It analyzes its benefits in the process of industrial integration. Finally, in the experiment and analysis part, a related experiment is designed to conduct a comprehensive analysis of the impact of the holding of sports events on the natural ecotourism of the city. In the analysis part, a detailed analysis and comparison of the specific effects after the industrial integration is carried out.

## Figures and Tables

**Figure 1:** Osmosis fusion mode.

**Figure 2:** The realization process of industrial integration.

**Figure 3:** Recombination fusion mode.

**Figure 4:** Sports extension industry.

**Figure 5:** The goal model of ecotourism to achieve sustainable development.

**Figure 6:** Thinking target system of ecotourism area.

**Figure 7:** Changes in the actual value and predicted value of tourism revenue after industry integration.

**Figure 8:** Changes in the actual and predicted value of the tourism environmental load rate after industry integration.

**Figure 9:** Changes in the actual value and predicted value of the tourism energy exchange rate after industry integration.

**Figure 10:** Attraction of tourists before and after industrial integration.

**Table 1:** Whether sports events have an impact on urban tourism.

	Select frequency	% of the total
Influential	9	75
Hard to say	3	25
Total	12	100

**Table 2:** Whether the impact of sports events on urban tourism is important.

	Select frequency	% of the total
Very important	5	41.7
More important	5	41.7
Generally important	1	8.3
Not so important	1	8.3
Total	12	100

**Table 3:** Contents of the impact of large-scale sports events on urban tourism.

	Select frequency	Total number of people	Ratio between options
Economic impact	10	83.3	26.3
Impact on hardware	6	50	15.8
Impact on software	7	58.3	18.4
Impact on structure	7	58.3	18.4
Impact on communication	8	66.7	21.1

**Table 4:** The impact of large-scale sports events on urban tourism economy.

	Select frequency	Total number of people	Ratio between options
Number of people grows	9	75	47.4
Increasing income	6	50	31.6
Employment increase	4	33.3	21.1

**Table 5:** The impact of large-scale sports events on the number of tourists.

	Select frequency	Total number of people	Ratio between options
Long term	2	16.7	16.7
Temporary	3	25	25
Hard to say	7	58.3	58.3

## Data Availability

No data were used to support this study.

## References

[1] Zhang M., Wang X., Ding Y. (2018). Flight responses of blue sheep in Ningxia helan mountain national nature reserve. *Folia Zoologica -Praha*.

[2] Baum J., Cumming G. S., De Vos A. (2017). Understanding spatial variation in the drivers of nature-based tourism and their influence on the sustainability of private land conservation. *Ecological Economics*.

[3] Dhami I., Deng J., Strager M. (2017). Suitability-sensitivity analysis of nature-based tourism using geographic information systems and analytic hierarchy process. *Journal of Ecotourism*.

[4] Xu L., Ao C., Mao B. (2020). Which is more important, ecological conservation or recreational service? Evidence from a choice experiment in wetland nature reserve management. *Wetlands*.

[5] Ibarra-Michel J. P., Velarde M., Ramos J. (2018). Community-based ecotourism management: the case of a cooperative in mazatlán, sinaloa, Mexico. *Czech Journal of Tourism*.

[6] Shi F., Weaver D., Zhao Y., Huang M. F., Tang T., Liu Y. (2019). Toward an ecological civilization: mass comprehensive ecotourism indications among domestic visitors to a Chinese wetland protected area. *Tourism Management*.

[7] Stone M. T., Nyaupane G. P. (2017). Ecotourism influence on community needs and the functions of protected areas: a systems thinking approach. *Journal of Ecotourism*.

[8] Bae H. (2017). Research direction of ecotourism as an indicator of cultural services. *Journal of the Korean Institute of Forest Recreation*.

[9] Lee T. H., Jan F. H. (2018). Ecotourism behavior of nature-based tourists: an integrative framework. *Journal of Travel Research: The International Association of Travel Research and Marketing Professionals*.

[10] Hurych E. (2017). Authenticity in the perspective of sport tourism: some selected examples. Physical culture and sport. *Studies and Research*.

[11] Carvache-Franco M., Segarra-Ona M., Carrascosa-Lopez C. (2019). Segmentation and motivations in eco-tourism: the case of a coastal national park. *Ocean & Coastal Management*.

[12] Salemi M., Jozi S. A., Malmasi S., Rezaian S. (2019). A new model of ecological carrying capacity for developing ecotourism in the protected area of the north karkheh, Iran. *Journal of the Indian Society of Remote Sensing*.

[13] Radkovic A. Z., Dongen W., Kirao L., Guay P. J., Weston M. A. (2019). Birdwatchers evoke longer escape distances than pedestrians in some African birds. *Journal of Ecotourism*.

[14] Retka J., Jepson P., Ladle R. J. (2019). Assessing cultural ecosystem services of a large marine protected area through social media photographs. *Ocean & Coastal Management*.

[15] Dupke C., Dormann C. F., Heurich M. (2019). Does public participation shift German national park priorities away from nature conservation?. *Environmental Conservation*.

[16] Cohen-Hattab K., Gelbman A., Shoval N. (2018). From ideological space to recreational tourism: the Israeli forest. *Journal of Tourism and Cultural Change*.

[17] Amis L. (2017). Mega-sporting events and human rights—a time for more teamwork?. *Business & Human Rights Journal*.

[18] Rojas-Mendez J. I., Davies G., Jamsawang J., Duque J. L. S., Pipoli G. M. (2019). Explaining the mixed outcomes from hosting major sporting events in promoting tourism. *Tourism Management*.

[19] Ireland R., Bunn C., Reith G. (2019). Commercial determinants of health: advertising of alcohol and unhealthy foods during sporting events. *Bulletin of the World Health Organization*.

[20] Azzali S. (2019). Challenges and key factors in planning legacies of mega sporting events: lessons learned from London, Sochi, and Rio de Janeiro. *Archnet-IJAR: International Journal of Architectural Research*.

[21] Mcgillivray D., Mcpherson G., Misener L. (2018). Major sporting events and geographies of disability. *Urban Geography*.

[22] Kan F., Takuya F., Hiroaki F. (2017). An examination of the relationship between spectating intention or behavior at sporting events, and place attachment: the case of imabari football club. *Journal of Japan Society of Sports Industry*.

[23] Bonasso P., Lucke-Wold B. P., Riffon M., Long D., Wilson A., Knight J. (2017). The effect of sporting events on medical transport time at a level 1 trauma center: a retrospective cohort study. *West Virginia Medical Journal*.

